The article "Investigating Feature Ranking Methods for Sub-Band and Relative Power Features in Motor Imagery Task Classification" was published in 2021. Journal: J Healthc Eng.

# Investigating Feature Ranking Methods for Sub-Band and Relative Power Features in Motor Imagery Task Classification

**DOI:** 10.1155/2021/3928470

**Published:** 2021-09-27

**Authors:** Samrudhi Mohdiwale, Mridu Sahu, G. R. Sinha, Humaira Nisar

**Affiliations:** ^1^National Institute of Technology Raipur, Raipur, India; ^2^Myanmar Institute of Information Technology, Mandalay, Myanmar; ^3^Universiti Tunku Abdul Rahman, Kampar, Malaysia

## Abstract

Interpreting the brain commands is now easier using brain-computer interface (BCI) technologies. Motor imagery (MI) signal detection is one of the BCI applications, where the movements of the hand and feet can be recognized via brain commands that can be further used to handle emergency situations. Design of BCI techniques encountered challenges of BCI illiteracy, poor signal to noise ratio, intersubject variability, complexity, and performance. The automated models designed for emergency should have lesser complexity and higher performance. To deal with the challenges related to the complexity performance tradeoff, the frequency features of brain signal are utilized in this study. Feature matrix is created from the power of brain frequencies, and newly proposed relative power features are used. Analysis of the relative power of alpha sub-band to beta, gamma, and theta sub-band has been done. These proposed relative features are evaluated with the help of different classifiers. For motor imagery classification, the proposed approach resulted in a maximum accuracy of 93.51% compared to other existing approaches. To check the significance of newly added features, feature ranking approaches, namely, mutual information, chi-square, and correlation, are used. The ranking of features shows that the relative power features are significant for MI task classification. The chi-square provides the best tradeoff between accuracy and feature space. We found that the addition of relative power features improves the overall performance. The proposed models could also provide quick response having reduced complexity.

## 1. Introduction and Background

Brain activates the sensory motor rhythm for virtual motor movements such as hand or feet; however, the actual motor movement of the body parts is not essential. The activation properties of brain correlate the activities with the motor movements, which help in different emergency situations to provide quick response in the system [1, 2]. Amyotrophic lateral sclerosis (ALS) is one of the serious diseases of brain, where the patient loses their control over the body and only the mind is active. The brain-computer interface (BCI) technology designed for motor imagery task can assist the patients in communication [3]. BCI technology enables the translation of brain commands of motor actions to read the brain signal and thus is considered as effective method for providing faster and accurate response [4, 5]. The accuracy of BCI is very sensitive to internal and external noises, intersubject variabilities, and nonstationarity and nonlinearity of brain signal. Also, when BCI models are considered, the performance is limited by the algorithm simplicity.

The article "Investigating Feature Ranking Methods for Sub-Band and Relative Power Features in Motor Imagery Task Classification" was published in 2021. Journal: J Healthc Eng.

The structure of brain consists of four lobes, which are frontal, parietal, occipital, and temporal lobe. Each lobe is responsible for a specific task. Frontal lobe is active when emotion, problem solving, speech, and movement related tasks are performed; and the parietal lobe is responsible for sensation, taste, speech, reading, and so forth. Occipital lobe is responsible for vision, visual stimuli, and interpretation. The temporal lobe is related to hearing, comprehension of language, and information retrieval. The movement related actions are performed by the motor cortex which is located in back part of the frontal lobe almost in the center of brain. Thus, the signal received from the motor cortex from the frontal and parietal lobes is helpful in understanding and classifying motor imagery actions [6].

Numerous studies are reported in the literature to recognize and interpret the brain signals. The motor imagery commands are decoded using Fourier transform, short time Fourier transform, common spatial pattern and its variants, local mean decomposition, wavelet packet decomposition, and power spectral density [5, 7–11]. Wavelets are used for various applications such as denoising, feature extraction, and frequency sub-band categorization [12, 13]. Band power is also one of the widely used features. Brodu et al. [14] presented a comparative study on band power extraction for motor imagery (MI) task in which periodogram, autoregression, Butterworth filter, spectrogram, and Morlet wavelets are evaluated and wavelets are recommended for obtaining satisfactory results. Wang et al. [15] evaluated time frequency representation synthesis for spatial filters. Qin and He [16] developed wavelet and event-related desynchronization-based method for MI task classification, in which further comparison is based on the weighted energy difference of electrode pairs for MI task. Kim et al. [17] proposed an optimal channel based feature extraction via difference weighted power spectral density for MI task classification. The single session and session-to-session accuracies were evaluated for reliability of the proposed model. Tidare et al. [18] studied a single limb hand open and close movement by power measures. Linear regression and convolution neural network (CNN) are used to evaluate the performance and CNN was found to be outperforming. However, it still suffers from less accuracy, nearly 60% for the used dataset. This shows the chances of improvement via deep learning with higher variety of datasets. Mu-beta rhythms were proved efficient; however, to enhance the training feedback, SSVEP based hybrid BCI is proposed in [19]. Further studies also reported combination of EEG from motor and somatosensory cortex together for improving the performance of BCI [20]. Discriminative feature learning, sliding window common spatial patterns are some recent approaches used for MI task classification [21, 22]. EEG-Net with Temporary Constrained Sparse Group Lasso also proves its efficiency in MI task classification [23]. Akbulut et al. [24] proposed alpha and beta frequency power for MI task classification as the frequency represented as most responsible frequency of motor tasks. The performance evaluation is based on nearest neighbor, SVM, logistic regression, naïve Bayes, and decision tree classifiers. From these studies, decision tree and random forest are reported as the most widely used classifiers for MI task classification and, thus, in the current study, we have taken them into consideration. Deep learning is a widely accepted area nowadays, but the computational cost, complexity of model, and lack of sufficient data still create implementation challenges.

The article "Investigating Feature Ranking Methods for Sub-Band and Relative Power Features in Motor Imagery Task Classification" was published in 2021. Journal: J Healthc Eng.

### 1.1. Motivation and Objectives

Motor imagery task classification is one of the open challenging tasks for which various methods are proposed. Common spatial pattern (CSP) and its variants show the improved accuracy for MI task classification, but these are sensitive to noise; and the spectral and temporal characteristics of signals are neglected. Moreover, the variants are susceptible to channel specific data. To mitigate these limitations, frequency-based features are gaining popularity nowadays. Keeping in mind the popularity of frequency specific features, the current study aims to

1. Improve the performance of motor imagery task classification using frequency-based features
2. Analyze the relative power of frequency for classification of motor imagery task
3. Maintain the tradeoff between accuracy and feature space for minimal complexity of the model

The rest of the paper is organized as follows.  Section 2 presents the methodology for the process adopted to improve the performance of motor imagery task classification.  Section 3 provides the details of the results obtained from different classifiers.  Section 4 provides the detailed discussion on the results and Section 5 concludes the paper with future aspects in the area.

The article "Investigating Feature Ranking Methods for Sub-Band and Relative Power Features in Motor Imagery Task Classification" was published in 2021. Journal: J Healthc Eng.

## 2. Methodology

In this section, the details of the method incorporated to classify the motor imagery signal are described. First, the dataset used in the current work is described. Second, the features and feature extraction methods from brain signal used for MI task are discussed. Furthermore, feature ranking algorithms are used to evaluate the performance of newly added features.  Figure 1 represents the overall flow of processing involved in MI task classification.

In Figure 1, the processing of work accomplishes on EEG based MI task dataset. The description of the dataset is provided in Section 2.1. EEG signals are preprocessed using Butterworth filter and variety of features extracted from the wavelets of different power bands which are alpha, beta, gamma, and theta. To get the most significant feature and evaluate the suitability of feature ranking method, three different feature ranking methods, namely, mutual information, chi-square, and correlation, are performed. Classification on all feature sets and ranked feature set has been done using listed classification techniques. Results are evaluated based on accuracy, precision, recall, and F1-score. The results are also compared with existing techniques on the same dataset. Further details on each block of Figure 1 are presented further in the section.

### 2.1. Dataset Description

The current study utilizes an open source dataset available for MI task classification, which has been accessed from BNCI Horizon 2020 website. In this dataset, cue grazed recordings of 10 subjects in a single session of 8 runs, each of 20 trails, are available. The subjects were asked to perform hand and feet movements as per the cue. Participants had the task of performing sustained (5 seconds) kinesthetic motor imagery (MI) of the right hand and of the feet each as instructed by the cue. Feedback was presented in form of a white colored bar graph. The length of the bar graph reflected the amount of correct classifications over the last second. EEG was measured with a biosignal amplifier and active Ag/AgCl electrodes at a sampling rate of 512 Hz. The electrodes placement was designed for obtaining three Laplacian derivations. To record the EEG signals, wet electrodes were fixed at central lobe, that is, C3, C4, and Cz [25, 26]. In this experiment, we have used 5-fold cross-validation throughout the work. Although there are different datasets available for MI task classification, this dataset has been chosen, since it provides a large number of data samples along with the different subjects available for recording with reduced intersubject variability issue.

The article "Investigating Feature Ranking Methods for Sub-Band and Relative Power Features in Motor Imagery Task Classification" was published in 2021. Journal: J Healthc Eng.

### 2.2. Signal Preprocessing

The signals obtained from the source electrode contain artifacts such as undesired frequencies which are removed by preprocessing the data using Butterworth band-pass filter of 5th order having a passband frequency of 0.5 Hz and stopband frequency of 100 Hz. The filter transfer function is given in (1) [27]. Maximally flat response and uniform passband property make the filter more suitable for preprocessing of brain signals.

### 2.3. Feature Extraction

Feature extraction is an important step to reduce the dimensionality of a signal and simultaneously extract the important information. EEG recordings consist of large oscillations of different frequencies and various studies on brain oscillatory frequencies reflect the event-related synchronization and desynchronization in alpha, beta, and gamma rhythms [28]. Power spectral density (PSD) of these frequencies helps to analyze the impact of signal while performing MI task. Since the results from different studies suggest that only average power of these features is not sufficient to discriminate hand and feet movement, relative power and variance of the PSD are proposed in the current study for analysis.

To obtain the oscillations of different frequencies from EEG signal, discrete wavelet transform (DWT) of 5th level decomposition and “dB4” wavelet are used. The technique localizes the changes in frequency of signal over time and thus both time information and frequency information are taken into consideration unlike CSP features with reduced computational complexity. In wavelet transform, the signal is downsampled by 2 and up to 5 levels, and, using downsampling, we get 5 detailed coefficients and 1 approximate coefficient. The 5th level DWT has been chosen because its decomposition provides the range of frequencies distributed similar to brain oscillatory frequencies. The “dB4” is chosen based on the effective results from different studies [17, 18, 29]. The frequency ranges for the coefficients are as follows: D1: 50–100 Hz (called noise and rejected), D2: 25–50 Hz (gamma), D3: 12.5–25 Hz (beta), D4: 6.25–12.5 Hz (alpha), D5: 3.125–6.25 Hz (theta), and A5: 0–3.125 Hz (delta, none of our interest).

In the current work, average power and relative and varied powers from each frequency band of interest are used as a new feature combination which can effectively distinguish the MI task. In Figure 2, it can be seen that the average as well as variance of each oscillatory frequency can play a major role. While the concept of relative power is considered here because the event-related synchronization and desynchronization between alpha, beta, and gamma rhythm are used for the MI task to happen, this will add extra efficient features for MI task classification. Average power of each frequency and variance of power distribution are obtained by using signal reconstruction corresponding to the wavelet coefficients of alpha, beta, and gamma. Pwelch function of MATLAB is used for the calculation of power spectral density, and the feature matrix is as follows: [*A*_11_, *A*_12_, *A*_11_, *A*_13_, *A*_14_, *A*_15_, *A*_16_, *A*_17_, *A*_18_, *A*_19_, *A*_110_, *A*_111_,  *A*_111_], where *A*_11_ −  *A*_14_ denote average powers of alpha, beta, gamma, and theta band, respectively, *A*_15_ −  *A*_17_ denote relative powers of alpha to beta, gamma, and theta band, respectively, and *A*_18_ −  *A*_111_ denote varied powers of alpha, beta, gamma, and theta band, respectively. The algorithm used in the current study is presented as Algorithm 1.

The article "Investigating Feature Ranking Methods for Sub-Band and Relative Power Features in Motor Imagery Task Classification" was published in 2021. Journal: J Healthc Eng.

The obtained feature matrix has dimension of 1 × 11 for each trial from the dataset. The overall feature matrix of size 1260 × 11  is obtained. To evaluate the significance of features, feature ranking method is used and comparative analysis is carried out. In the next section, feature ranking method is described in detail.

### 2.4. Feature Ranking

Feature ranking methods help in evaluating the importance of the proposed features which are used in the work. These methods will provide rank of features based on different methods. Mutual information, chi-square (*χ*2), and correlation are the most widely used feature ranking methods. In this study, these three techniques are used to find the most as well as least important features. The details of the method are discussed below.

#### 2.4.1. Mutual Information

Mutual information provides the measure of dependency between features and can be obtained by

(1) $$\begin{array}{c} I\left(A,B\right)=\sum_{A}\sum_{B}p\left(A,B\right)\log\frac{p\left(A,B\right)}{p\left(A\right)p\left(B\right)}\;, \end{array}$$

where A and B are two different features, respectively; *p*(*A*, *B*) is the joint probability; *p*(*A*) and *p*(*B*) are individual probabilities and *I*(*A*, *B*) denotes the mutual information between two features. The higher the mutual information is, the higher the dependency is; hence, features having higher mutual information will be ranked higher than others [30, 31].

#### 2.4.2. Chi-Square Method

Chi-square method of feature selection ranks the features based on the dependency of features on the respective class. We are interested in features which are highly dependent on the class and this method gives the higher rank to the feature which is more dependent on class than others. These feature frequencies are calculated from each sample. Null hypothesis for the test is formulated as the features are highly dependent with an alternative hypothesis as the features are independent. The value of *χ*2 is calculated by using the following formula [30, 32]:

(2) $$\begin{array}{c} \chi 2=\;\frac{{\left(F_{O}-F_{E}\right)}^{2}}{F_{E}}, \end{array}$$

where *F*_O_ is the observed frequency of dependent features and *F*_*E*_ is the expected frequency of the dependent features. Alpha (confidence interval) is chosen as 0.05.

The article "Investigating Feature Ranking Methods for Sub-Band and Relative Power Features in Motor Imagery Task Classification" was published in 2021. Journal: J Healthc Eng.

#### 2.4.3. Correlation Method

Correlation measure provides a method to identify highly correlated features of the data. Higher correlation signifies the lesser generalizability of the model. Hence, these features need to be removed to reduce the dimension and to improve the generalizability of the selected classifier. The correlation is calculated using the following formula [30, 33]:

(3) $$\begin{array}{c} r=\frac{k\left(\sum AB\right)-\left(\sum A\right)\left(\sum B\right)}{\sqrt{\left[\left(\sum A^{2}\right)-\left(\sum A\right)\right]\left[k\left(\left(\sum B^{2}\right)-\sum B\right)\right]}}, \end{array}$$

where *A* and *B* are two features from the set of features and *r* denotes the correlation coefficient between features. The correlation between more than two features can be visualized in heat map. In this map, highly correlated features are darker, while the features having lesser correlation show less intensity of the color. From the heat map, one can rank the highly positively or negatively correlated features [30, 33].

### 2.5. Classification and Comparative Analysis

The feature matrix obtained using the method is fed into different classifiers to evaluate the performance of features. Five well-known classifiers, namely, decision tree (DT), fine k-nearest neighbor (KNN), weighted KNN (WKNN), quadratic support vector machine (QSVM), and random forest, are used for classification. The results obtained from classification are shown and discussed in Section 3. The results obtained after classification are analyzed based on the classification accuracy of classifier, precision, recall, and F1-score [34]. The comparative analysis of the current study with different existing approaches is also presented in the next section.

## 3. Results and Discussion

The experiment was performed on a system configuration of Intel Core *i*5 processor and 8 GB RAM. Open source dataset of motor imagery task classification is evaluated with the proposed approach and compared with different existing approaches. The results obtained from the current study are presented in this section.

### 3.1. Results of Different Classifiers without Feature Ranking

In this study, five classifiers are used for classification of MI tasks and the results obtained are shown in Table 1. Five of the most widely used classifiers are chosen for the study, which are decision tree, fine KNN, weighted KNN, quadratic SVM, and random forest.

The article "Investigating Feature Ranking Methods for Sub-Band and Relative Power Features in Motor Imagery Task Classification" was published in 2021. Journal: J Healthc Eng.

Decision tree takes the decision based on experience by splitting the data and it works like a human brain. KNN is based on nearness criteria; that is, the lower the distance, the higher the chances of data to lie in that class. SVM creates a hyperplane to classify the objects. Random forest consists of multiple small decision trees on a random subset of data, and each tree will act as an expert to take the decision of split [34].

From the results, it is clear that, except SVM, all classifiers provide competitive accuracy. The highest accuracy obtained from the weighted KNN classifier is 93.51%.

Precision, recall, and F1-score measures are also important criteria while evaluating the performance of classifiers. The higher the precision is, the lower the number of false positive errors committed by the classifier is. Classifiers with large recall have very few positive examples misclassified. F-measure represents a harmonic mean between recall and precision. A high value of F-measure ensures that both precision and recall are reasonably high [34]. The precision, recall, and F1-scores of different classifiers are shown in Figure 3.

In Figure 3, it can be seen that, for values of precision, recall, and F1-score for classifiers ranging from 0.75 to 0.95, in decision tree, fine KNN, and random forest, we get outlier values; however, weighted KNN and QSVM does not have outliers. In weighted KNN, maximum values are above the 1st quartile range and have significant score of more than 0.85 which can be termed as good precision, recall, and F1-scores for MI task classification. Fine KNN also shows better values but has less accuracy than weighted KNN. Hence weighted KNN is used further in the study.

Feature ranking methods are evaluated for analysis in order to understand the role of power features. The detailed results on the ranking method are provided in the subsequent section.

### 3.2. Results of Different Classifiers with Feature Ranking Methods

Analysis of features is essential and crucial step to obtain the dominant features and reduce the dimensionality. As feature ranking can provide the relevant set of features, it also helps to reduce the overfitting and improve the generalizability of the classification model. This section discusses the results of different methods of feature ranking in detail.

#### 3.2.1. Results of Feature Ranking with Mutual Information

Mutual information is a very prominent method of feature ranking. The detailed method was discussed in Section 2.4.1. To obtain the results of feature ranking, the method is evaluated 10 times and the ranking obtained after each iteration is stored. Mutual information shows the dependency of features with respect to class. The higher the mutual information, the higher the significance of the feature.

The article "Investigating Feature Ranking Methods for Sub-Band and Relative Power Features in Motor Imagery Task Classification" was published in 2021. Journal: J Healthc Eng.

Top 6 features are selected out of 11 which are obtained from 10 iterations for all ten subjects.  Figure 4 represents the ranking of features obtained with the mutual information method. From Figure 4, it is clear that features {5, 7, 8, 10, 11} are the most valuable features, out of which 5 and 7 are relative power features and the others are varied power features. It can be seen that mutual information method of feature selection selects the variety of features containing alpha, theta, and gamma band.

#### 3.2.2. Results of Feature Ranking with Chi-Square Method

Chi-square test is performed for the ranking of features. The higher dependence of features on the class is preferred for ranking. Chi-square test rankings for 11 features are shown in Figure 5.

Chi-square method is another popular approach of feature selection. This method focuses on two values named F-Score and *P* values. The higher F-Score and the lower *P* values are the most significant features. In the current work, the same procedure is followed and top five features out of eleven are selected by the rank provided by chi-square method. The feature selection is performed for 10 iterations and the results are presented in Figure 5. Top five features are selected based on occurrence of features in multiple iterations. Feature set {6, 8, 9, 10, 11} is selected as most significant feature for further analysis.

#### 3.2.3. Results of Feature Ranking with Correlation Measure

The correlation method is another measure for feature ranking, which provides information of mutually correlated features. The heat map for the features of the ten subjects is shown in Figure 6.

In the heat map, darker color shows higher correlation, while lighter color has less correlation among the features. The correlated pairs obtained after 10 iterations of the correlation feature selection module are shown in 7.

Figure 7 shows the correlated pairs of feature. The higher the correlation, the lower the importance of feature; hence, feature {3, 7, 8, 9, 10, 11} can be discarded and accuracy can be calculated among the rest of the features for further analysis. From this, it can also be seen that there is no correlation among the features of relative power, that is, feature {5, 6}. This represents the significance of relative power features with respect to the correlation among them.

The article "Investigating Feature Ranking Methods for Sub-Band and Relative Power Features in Motor Imagery Task Classification" was published in 2021. Journal: J Healthc Eng.

#### 3.2.4. Overall Analysis of Feature Ranking Method on Accuracy

In this section, the overall analysis of the impact of relative and varied power on accuracy for MI task classification is presented. The accuracy has been calculated by considering the best features obtained from feature ranking method. The results are shown in Table 2.

When all features are taken into consideration, the average accuracy of 93.51% has been obtained, which is a significant result. We analyze the importance of relative power features by calculating the accuracy without considering them. The results show that, for six out of ten subjects, the accuracy is reduced and, for the rest of the subjects, there is a slight change in the accuracy, nearly ±0.2 to 0.6%, which is very small. Further, in the analysis, the best features from different ranking algorithms are selected based on the rank and the rest of the features are dropped out. The results for dropout of those features do not have more impact on the classification accuracy. In the subsequent section, a comparative analysis of different existing models and feature ranking methods is presented.

### 3.3. Comparative Analysis

To compare the proposed method with existing models, a comparative analysis is presented in this section. The results for comparison are based on the research papers using the same datasets [25, 26]. The proposed approach is compared with the most widely used feature, that is, CSP for MI task classification. The comparative results are shown in Figure 8. From the figure, it is clear that the average and varied power features with RF classifier outperform the CSP feature for most of the subjects. The figure also represents that the performance of CSP method is varied with the subjects, but our proposed approach does not have this issue. This ensures that the performance of the proposed approach mitigates the challenge related to intersubject variability.

Apart from the results presented in this dataset, some other studies reported performance for a few subjects. Sahu et al. reported the average performance of 60.5% for 3 subjects using principal component analysis [35]. In another study, M. Sahu and S. Shukla used a feature selection approach for improved classification of MI signals. In this study, an average accuracy of 58.25% for 4 subjects is reported [36]. Kumar and Sahu proposed PSO based analysis for MI task classification and this resulted in the highest accuracy achieved which is 68.75% [37]. To analyze the performance of feature ranking approach, we further evaluate the average loss of features and accuracy for different feature raking approach.

Figure 9 represents the loss or reduction in accuracy for different methods. If we select top 5 features from the feature set and calculate the accuracy, the variation in accuracy with existing accuracy of particular subject is termed as loss in accuracy. The higher the loss, the lower the significance of method. Correlation method shows the highest loss in accuracy with respect to accuracy of all the features. Mutual information method shows significant loss in accuracy, while chi-square method provides minimum loss in accuracy. So, chi-square method can be used to maintain the tradeoff if higher complexity is the issue.

The article "Investigating Feature Ranking Methods for Sub-Band and Relative Power Features in Motor Imagery Task Classification" was published in 2021. Journal: J Healthc Eng.

Further, in this study, to know the effect of dropout features with respect to accuracy, Figure 10 highlights the change in accuracy.

From Figure 10, it is clear that the highest accuracy is obtained by considering all eleven features. In mutual information, top six features are selected and accuracy of 93% is achieved, whereas, in chi-square method, top five features are selected and accuracy of 93.5% is obtained. In correlation method, top 5 features are selected but accuracy drastically reduces to 91.5%. Hence, it can be concluded that, in mutual information method and chi-square method, the tradeoff between feature space and accuracy is maintained.

## 4. Discussion

In the current study, the impact of relative power and variance of power is taken into consideration for classification of MI tasks. Signals obtained from brain are taken using electrodes placed on the motor cortex; hence, the study is based on frequency and power of signal from the motor cortex, that is, C3, C4, and Cz and nearby electrodes. To analyze the impact, different strategies are adopted. Ten subjects are considered for the evaluation of the proposed method for MI task classification. The results show that the proposed approach outperforms CSP based approach for classification; the reason behind this is the nature of frequency-based features which allows holding significant characteristics for each task efficiently. Overall average accuracy obtained in the study is 93.51%, which is consistent for all subjects, not like other approaches having higher accuracy for a few subjects. As an analysis of feature ranking method, the mutual information-based method delivers an average classification accuracy of 93.05% for the feature set {5, 7, 8, 10, 11}. In this method, the relative power features and varied power features show their significance with the slightest loss in accuracy. In the chi-square method, the analysis provides accuracy of 93.4% on the feature set {6, 8, 9, 10, 11}. In this method, the dominance of varied power feature is indicated, but it also shows the contribution of relative power feature of alpha to gamma ratio (6th feature). In correlation-based method, again the feature {5, 6} shows the least correlation. Hence, these proposed features are significant not only in the aspect of accuracy enhancement but also in different scenarios considered having mutual information and correlation of features as major concerns. The analysis also shows that the combination of features exhibits the tradeoff between accuracy and complexity of feature space when complexity is a major concern.

The article "Investigating Feature Ranking Methods for Sub-Band and Relative Power Features in Motor Imagery Task Classification" was published in 2021. Journal: J Healthc Eng.

## 5. Conclusion

The improvement in motor imagery based BCI is important in its sophisticated model and analysis. In the current study, MI signals are classified by the power of alpha, beta, and gamma frequencies along with the relative power. Five different classifiers are adopted to choose the better results from the variety of classifiers. The results of the classification suggest that all classifiers have competitive results but, based on accuracy, weighted KNN outperforms all the other classifiers. The proposed approach also outperforms the CSP-based feature extraction method for the given dataset. The proposed approach not only resolves the problem to maintain the tradeoff and complexity but also mitigates the intersubject variability problem. To judge the significance of new added features, feature ranking method is presented. Based on the mutual information, chi-square, and correlation methods of feature ranking, results are calculated and compared. The results of the feature ranking method suggest that when feature space and time complexity are the concerns, then chi-square method outperformers other feature ranking methods with reduction of 45% feature space. However, when the accuracy of the method is concerned for BCI, the addition of relative power feature improves the overall performance of the system. Future era will be based on BCI, which flourishes the scope of further research to meet the challenges of electrode placements and selection, signal to noise ratio improvement, and device dependency reduction.

## Figures and Tables

**Figure 1:** Flowchart of the proposed method.

**Figure 2:** Power spectral density of different brain oscillatory frequencies.

**Figure 3:** Precision, recall, and F1-scores for different classifiers.

**Figure 4:** Feature ranking with mutual information.

**Figure 5:** Feature rankings with chi-square method.

**Figure 6:** Heat map of all ten subjects for correlated and uncorrelated features.

**Figure 7:** Correlated pairs of features.

**Figure 8:** Comparison of the proposed approach with the existing approaches.

**Figure 9:** Average loss in accuracy for implemented methods of feature ranking.

The article "Investigating Feature Ranking Methods for Sub-Band and Relative Power Features in Motor Imagery Task Classification" was published in 2021. Journal: J Healthc Eng.

**Figure 10:** Change in accuracy with feature ranking algorithms.

**Algorithm 1:** Algorithm for the proposed approach.

**Table 1:** Classification accuracy of different classifiers.

Subjects	Classification accuracy (in %)				
	Tree	Fine KNN	Weighted KNN	Quadratic SVM	Random forest
S01	89.1	92.9	94.3	65.3	89.4
S02	87.3	91.9	92.8	70.5	91.1
S03	89.5	92.9	94.2	71	91.34
S04	88.2	90.6	93.6	67.3	90.625
S05	85.5	91.8	93.1	66.1	86.77
S06	87.7	90.2	93.1	58.4	90.86
S07	88.7	89.1	91.6	69	87.01
S08	86.7	91.3	92.9	64.4	89.66
S09	**92**	92.7	95.2	**73.7**	**92.78**
S10	87.7	**92.9**	94.3	67.5	91.34
AVG	88.24	91.63	**93.51**	67.32	90.0885

Bold letters show the maximum classification accuracy of the classifier.

**Table 2:** Analysis of accuracy (in %) for impact of relative and varied power features.

Subjects	Accuracy with all features	Accuracy without relative power features	Accuracy with best features from mutual information method	Accuracy with best features from chi-square method	Accuracy with dropping out correlated features
S01	94.3	**94.9**	93.8	94.2	92.4
S02	92.8	93	**93.7**	93.1	92.5
S03	94.2	93.3	93.2	**94.2**	90.4
S04	**93.6**	91.9	92.1	**93.6**	91.7
S05	**93.1**	92.5	92.6	**93.1**	91.8
S06	**93.1**	92.7	92.3	**93.1**	90.1
S07	91.6	91.4	**91.7**	91.6	89.7
S08	92.9	92.6	92.2	**93.01**	90.6
S09	95.2	**95.4**	**95.4**	95.2	91.7
S10	94.3	**94.9**	93.8	94.3	92.1

Bold letters show the maximum classification accuracy of the classifier.

## Data Availability

Publicly available datasets are used in this research, which can be accessed via http://bnci-horizon-2020.eu/database/data-sets.
